This article has been retracted.

# Superparamagnetic iron oxide nanoparticles conjugated with Aβ oligomer-specific scFv antibody and class A scavenger receptor activator show therapeutic potentials for Alzheimer’s Disease

**DOI:** 10.1186/s12951-020-00723-1

**Published:** 2020-11-07

**Authors:** Xiao-ge Liu, Lun Zhang, Shuai Lu, Dong-qun Liu, Ya-ru Huang, Jie Zhu, Wei-wei Zhou, Xiao-lin Yu, Rui-tian Liu

**Affiliations:** 1 State Key Laboratory of Biochemical Engineering, Institute of Process Engineering, Chinese Academy of Sciences, Beijing, 100190 China; 2 School of Chemical Engineering, University of Chinese Academy of Sciences, Beijing, 100049 China

**Keywords:** Alzheimer’s disease, β-Amyloid, Oligomer, Class A scavenger receptor, Therapy

## Abstract

**Background:**

Alzheimer’s disease (AD) is a progressive neurodegenerative disorder. No disease-modifying strategy to prevent or delay AD progression currently exists. Aβ oligomers (AβOs), rather than monomers or fibrils, are considered as the primary neurotoxic species. Therapeutic approaches that direct against AβOs and promote Aβ clearance may have great value for AD treatment.

**Results:**

We here reported a multifunctional superparamagnetic iron oxide nanoparticle conjugated with Aβ oligomer-specific scFv antibody W20 and class A scavenger receptor activator XD4 (W20/XD4-SPIONs). Besides the diagnostic value, W20/XD4-SPIONs retained the anti-Aβ properties of W20 and XD4 by inhibiting Aβ aggregation, attenuating AβO-induced cytotoxicity and increasing microglial phagocytosis of Aβ. When applied to APP/PS1 mice, W20/XD4-SPIONs significantly rescued cognitive deficits and alleviated neuropathology of AD mice.

**Conclusion:**

These results suggest that W20/XD4-SPIONs show therapeutic benefits for AD. In combination with the early diagnostic property, W20/XD4-SPIONs present as a promising agent for early-stage AD diagnosis and intervention.

## Background

Alzheimer’s disease (AD) is the most common neurodegenerative disorder, which is characterized by progressive memory loss and cognitive decline. The pathological hallmarks of AD are the presence of extracellular β-amyloid (Aβ) plaques and intraneuronal neurofibrillary tangles aggregated from the microtubule-associated protein tau [1]. The prevalence of AD is increasing, which causes heavily social and economic burden over the world. Despite decades of efforts to understand AD pathophysiology and to develop therapies, effective strategies to prevent and cure it remain elusive [2].

The amyloid cascade hypothesis suggests that Aβ oligomers (AβOs), rather than monomers or insoluble fibrils, are the primary toxic species in the pathogenesis of AD [3]. AβOs appear in the brains of AD patients decades before the onset of clinical symptoms [4–6], suggesting their potential use as a more appealing target than plaques at the early stage of AD. Moreover, mounting of evidences support a pivotal role of AβOs in neuronal dysfunction and synapse loss in AD [7–9]. AβOs bind to the plasma membranes of neuronal cells, trigger transmembrane signaling and abnormal intracellular changes, which lead to synapse failure and ultimately cognitive impairment [10]. Intensive efforts have been directed against AβOs. The antibodies targeting these oligomers are producing encouraging results although all of the antibodies against Aβ monomers did not show clinical efficacy in AD patients [3]. The Biologics License Application of aducanumab, a specific anti-AβOs antibody, has been submitted to FDA after the significant therapeutic efficacy in phase III clinical trials was obtained [11].

Compared with the full-effector Aβ-targeting antibodies, AβO-specific single-chain variable fragment (scFv) antibody may show promise in treating AD due to lack of Fc fragment, which would avoid inflammatory response and other potential side effects. In previous studies, we reported that an oligomer specific scFv antibody W20, which specifically bound to toxic AβOs and inhibited their neurotoxicity with high safety [12–14]. W20 significantly attenuated memory deficits and Aβ burden in AD transgenic mice. However, W20 showed low efficiency in AβOs clearance. To resolve such problem, we introduced an heptapeptide XD4 in combination with W20. XD4 peptide was isolated from a Ph.D.-C7C library by phage display, which can activate the class A scavenger receptor (SR-A) on the microglia and promote AβOs phagocytosis [15]. Here, we conjugated W20 and XD4 onto superparamagnetic iron oxide nanoparticles (SPIONs) to construct novel multifunctional nanoparticles, W20/XD4-SPIONs. We previously demonstrated that W20/XD4-SPIONs, as an AβO-targeted molecular MRI contrast probe, exhibited early diagnostic potentials for AD [16]. Moreover, W20/XD4-SPIONs showed the properties of good biocompatibility, high stability and low cytotoxicity. In this study, we investigated whether W20/XD4-SPIONs retained the dual anti-Aβ functions of W20 and XD4 in vitro, and assessed their effects on cognitive performance and neuropathology in APP/PS1 mouse model.

## Results

### The characterization of W20/XD4-SPIONs

W20/XD4-SPIONs were constructed by conjugating W20 antibody and XD4 peptide onto the PEG-coated SPIONs (Fig. 1a). The conjugative efficiency of W20 and XD4 was 50% and 21.3%, respectively. Our Transmission electron microscopy (TEM) imaging demonstrated that W20/XD4-SPIONs were mono-dispersed with a mean diameter of 10.1 ± 1.5 nm (Fig. 1b, c). Dynamic light scattering (DLS) measurement demonstrated that the hydrodynamic diameters of the unconjugated-SPIONs and W20/XD4-SPIONs were 19.6 ± 2.5 nm and 28.7 ± 2.1 nm, respectively (Fig. 1d). W20/XD4-SPIONs showed a zeta potential of approximately − 29 mV.

**Fig. 1:** Characterization of W20/XD4-SPIONs. **a** Schematic illustration of W20/XD4-SPIONs. **b** The morphology of SPIONs and W20/XD4-SPIONs were imaged by TEM. Scale bar 50 nm. **c** The size distribution of SPIONs and W20/XD4-SPIONs detected by TEM. **d** The hydrodynamic diameters of SPIONs and W20/XD4-SPIONs were detected by DLS. **e** Cy7-labeled various SPIONs were injected to nude mice via tail vein with or without mannitol combination. The brains of mice were collected at 6 h post-injection, the Cy7 fluorescence signal was detected using IVIS spectrum imaging system.

To detect whether W20/XD4-SPIONs can cross the blood–brain barrier (BBB), Cy7-labeled various SPIONs were injected to nude mice via tail vein with or without mannitol combination. The mice were sacrificed after heart perfusion 6 h post-injection and their brains were collected for Cy7 fluorescence measurement. Pronounced fluorescence signal was observed in the brains of mice treated with all the tested SPIONs, suggesting that W20/XD4-SPIONs may readily penetrate BBB to reach the brain area. Moreover, the combination of mannitol significantly increased the BBB permeability of various SPIONs (Fig. 1e).

### W20/XD4-SPIONs inhibited Aβ aggregation and cytotoxicity and reduced the inflammatory cytokine production in vitro

In our previous studies, oligomer-specific antibody W20 and heptapeptide XD4 have been shown to inhibit Aβ aggregation, attenuate AβO-induced cytotoxicity and reduce the production of proinflammatory cytokines [12, 14, 15]*.* Here we investigated whether W20/XD4-SPIONs retained the anti-Aβ functions of W20 and XD4. In Aβ aggregation assay, Aβ42 alone showed the expected nucleation-dependent polymerization process, while both W20/XD4-SPIONs and W20-SPIONs significantly inhibited Aβ42 aggregation in a concentration-dependent manner, with a complete suppression at 1000 μg/mL (Fig. 2a). Similarly, 4 μM AβOs alone or combined with unconjugated-SPIONs caused a significant reduction in the viability of SH-SY5Y cells, whereas the addition of XD4-SPIONs, W20-SPIONs and W20/XD4-SPIONs increased cell viability by 41.2%, 44.1% and 52.9%, respectively (Fig. 2b). Furthermore, we detected the inflammatory cytokine production in BV-2 cells challenged by AβOs. The levels of IL-6 and TNF-α were elevated in AβO-treated cell supernatants, while W20/XD4-SPIONs resulted in a more significant reduction in these inflammatory factor levels than XD4-SPIONs and W20-SPIONs did (Fig. 2c, d). In the meanwhile, we determined the levels of inflammatory mediators such as iNOS and COX-2 in BV-2 cell lysates by western-blot (Fig. 2e). The results demonstrated that the levels of iNOS and COX-2 were all elevated by AβOs challenge but significantly decreased by W20/XD4-SPIONs treatment (Fig. 2f). These results indicated that W20/XD4-SPIONs significantly inhibited Aβ aggregation and cytotoxicity, as well as the inflammatory cytokine production in BV-2 cells. W20/XD4-SPIONs exhibited better effects than XD4-SPIONs and W20-SPIONs did.

**Fig. 2:** W20/XD4-SPIONs inhibited Aβ42 aggregation and cytotoxicity and reduced inflammatory factor production in vitro. **a** The aggregation kinetics of Aβ42 incubated with or without 100 or 1000 μg/mL W20-SPIONs or W20/XD4-SPIONs was assessed by thioflavin T fluorescence assay. **b** SH-SY5Y cells were treated with various SPIONs in the presence or absence of 4 μM AβOs for 48 h, the cell viability was determined by MTT assay. The levels of IL-6 (**c**) and TNF-α (**d**) in the supernatants of BV-2 cells treated with various SPIONs in the presence or absence of 4 μM AβOs for 12 h were determined using corresponding ELISA kits. **e** Western-blot analysis of iNOS and COX2 in the BV-2 cell lysates treated with various SPIONs in the presence of 4 μM AβOs or AβOs alone. **f** Quantification of iNOS and COX2 in (**e**). Data represent means ± SEM and were analyzed by one-way ANOVA with Tukey’s test (**b**,** c**, **d**, **f**) or two-way ANOVA with Dunnett’s test (**a**). *P < 0.05, **P < 0.01, ***P < 0.001

### W20/XD4-SPIONs rescued cognitive deficits in AD mice

After 28-day treatment of W20/XD4-SPIONs, we applied Y-maze test, Morris water maze (MWM) test and Novel object recognition test (NOR) to assess the effects of various SPIONs on the cognitive performance of AD mice (Fig. 3a). In Y-maze test, WT mice spent more time and showed more entries in the novel arm, whereas vehicle- or unconjugated SPIONs-treated AD mice had no preference for the novel arm (Fig. 3b, c). Compared with the AD control mice, AD mice treated with XD4-SPIONs, W20-SPIONs or W20/XD4-SPIONs showed significantly improved spatial memory by more residence time (Fig. 3b) and more entries (Fig. 3c) in the novel arm. Notably, W20/XD4-SPIONs exhibited the best effect on the memory retention in all tested groups. Consistently, in MWM test, AD mice treated with W20/XD4-SPIONs or W20-SPIONs took shorter time to reach the platform than vehicle-treated AD mouse controls during the acquisition period (Fig. 3d). In the probe trials, AD mice treated with XD4-SPIONs, W20-SPIONs or W20/XD4-SPIONs also exhibited spatially-oriented swimming behavior, shorter escape latencies (Fig. 3e), more times of platform crossing (Fig. 3f) and more time spent in the target quadrant (Fig. 3g) than vehicle- or unconjugated SPIONs-treated AD mice did. Moreover, no significant difference in the swimming speed of mice was observed within the mouse groups in the training period and the probe trials of MWM test, indicating that neither group was impaired in motility and exploratory activities. In object recognition test, vehicle- or unconjugated SPIONs-treated AD mice did not show any preference to the novel object, while AD mice treated with XD4-SPIONs, W20-SPIONs or W20/XD4-SPIONs exhibited a remarkable increase in investigation to the novel object (Fig. 3h). Collectively, these findings indicated that W20/XD4-SPIONs significantly attenuated cognitive deficits in AD mice, and exhibited the best effects among all of the tested SPIONs.

**Fig. 3:** W20/XD4-SPIONs rescued cognitive deficits in AD mice. **a** Schematic representation of pharmacological treatment and experimental measurement. **b**, **c** The short-term memory of AD mice and their WT littermates treated with various SPIONs was measured by Y-maze. The time spent in the novel arm (**b**) and the number of entries (**c**) were recorded. **d**–**g** Spatial learning and memory retention of AD mice and their WT littermates treated with various SPIONs were assessed using the Morris water maze. **d** During training trials, the latency to find the hidden platform was measured. During probe trials, the latency to the position of the removed platform (**e**), the number of platform crossings (**f**) and the time spent in target quadrant (**g**) were determined. (**h**) The object recognition test was performed in AD mice and their WT littermates treated with various SPIONs. The results were expressed as discrimination index. n = 8 mice/group. Data represent means ± SEM and were analyzed by one-way ANOVA with Tukey’s test (**b**, **c**, **e–h**) or two-way ANOVA with Dunnett’s test (**d**). *P < 0.05, **P < 0.01, ***P < 0.001

### W20/XD4-SPIONs reduced neuroinflammation in the brains of AD mice

The increased glial activation and inflammatory cytokine production cause neuroinflammation, which are strongly associated with AD onset and progression. We evaluated the gliosis in the brains of AD mice and their WT littermates by GFAP immunostaining (Fig. 4a) and Iba-1 immunostaining (Fig. 4b). The results showed that the immunostaining area of GFAP and Iba-1 were significantly decreased in the brains of AD mice treated with XD4-SPIONs, W20-SPIONs or W20/XD4-SPIONs. W20/XD4-SPIONs reduced GFAP-positive area in the cortex and hippocampus by 65.2% and 51.6%, respectively (Fig. 4c), and Iba-1-positive area by 64.1% and 79.6% (Fig. 4d) in the brains of AD mice, indicating that W20/XD4-SPIONs significantly attenuated astrocytosis and microgliosis in AD mouse brains.

**Fig. 4:** W20/XD4-SPIONs reduced neuroinflammation and oxidative stress in the brains of AD mice. GFAP immunostaining (**a**) and Iba-1 immunostaining (**b**) in the brains of AD mice treated with various SPIONs. Scale bar 250 μm. Quantification of GFAP (**c**) and Iba-1 (**d**) immunostaining. The levels of IL-1β (**e**), IL-6 (**f**), and TNF-α (**g**) in the brain lysates of AD mice and their WT littermates treated with various SPIONs were determined using corresponding ELISA kits. The levels of GSH (**h**), GSSG (**i**), GSH/GSSG ratio (**j**) and ROS (**k**) in the brain lysates of AD mice and their WT littermates treated with various SPIONs were determined using corresponding commercial kits. n = 8 mice/group. Data represent means ± SEM and were analyzed by one-way ANOVA with Tukey’s test. *P < 0.05, **P < 0.01, ***P < 0.001

To further assess the effects of various SPIONs on the inflammatory cytokine production, we determined the levels of IL-1β, IL-6 and TNF-α in the mouse brain lysates by ELISA assay. A significant decrease in the levels of these inflammatory cytokine was observed in the brains of AD mice treated with XD4-SPIONs, W20-SPIONs or W20/XD4-SPIONs. Among these, W20/XD4-SPIONs significantly decreased the levels of IL-1β by 41.7% (Fig. 4e), IL-6 by 50.1% (Fig. 4f), and TNF-α by 55.6% (Fig. 4g), respectively.

### W20/XD4-SPIONs increased glutathione level and reduced reactive oxygen species level in the brains of AD mice

Toxic AβOs lead to extensive oxidative stress in neuronal cells, which play a key role in AD pathogenesis. Oxidative stress occurs when free radical production exceeds antioxidant capacity. Overproduction of reactive oxygen species (ROS) may cause an imbalance in the cell redox environment, leading to lipid peroxidation or metabolic dysfunction [17]. Glutathione (GSH) is the smallest intracellular protein thiol molecule in the cells, which prevents ROS-induced cell damage by converting reduced GSH to oxidized state (GSSG), while GSH/GSSG ratio is considered as an ideal indicator for the oxidative stress level. We determined the levels of GSH, GSSG and ROS in the brain lysates of AD mice and their WT littermates treated with various SPIONs. The results showed that W20/XD4-SPIONs significantly increased GSH levels (Fig. 4h), decreased GSSG levels (Fig. 4i) and increased GSH/GSSG ratios (Fig. 4j) in AD mice. A significant decrease in ROS level was also observed in the brains of AD mice treated with W20/XD4-SPIONs (Fig. 4k). These findings indicated that W20/XD4-SPIONs significantly reduced the oxidative stress level in the brains of AD mice. Moreover, XD4-SPIONs and W20-SPIONs also resulted in an increased GSH/GSSG ratio and a decrease ROS level, but less effective than W20/XD4-SPIONs did.

### W20/XD4-SPIONs reduced Aβ burden in the brains of AD mice

We next evaluated Aβ burden in the brains of AD mice treated with various SPIONs. Aβ plaques in the mouse brains were detected by 6E10 immunostaining. Compared with the vehicle treatment, XD4-SPIONs and W20-SPIONs significantly reduced the plaque areas in the brains of AD mice, and W20/XD4-SPIONs treatment resulted in the lowest plaque burdens (Fig. 5a, b). The levels of soluble and insoluble Aβ in the mouse brain lysates were further determined by ELISA. All conjugated-SPIONs, including XD4-SPIONs, W20-SPIONs and W20/XD4-SPIONs significantly reduced the levels of insoluble Aβ40 and Aβ42 (Fig. 5c, d) in AD brains. W20/XD4-SPIONs also significantly reduced soluble Aβ42 levels in the brains of AD mice (Fig. 5e), while soluble Aβ40 levels didn’t reach the statistical difference by various SPIONs treatment (Fig. 5f). These results demonstrated that the treatment of W20/XD4-SPIONs reduced Aβ burden in the brains of AD mice.

**Fig. 5:** W20/XD4-SPIONs attenuated Aβ pathology in the brains of AD mice. **a** 6E10 immunostaining for plaques in the brains of AD mice treated with various SPIONs. Scale bars 400 μm. **b** Quantification of Aβ-immunostaining areas in (**a**). The levels of insoluble Aβ40 (**c**), insoluble Aβ42 (**d**), soluble Aβ42 (**e**) and soluble Aβ40 (**f**) in the brain lysates of AD mice and their WT littermates treated with various SPIONs were detected by ELISA. n = 8 mice/group. Data represent means ± SEM and were analyzed by one-way ANOVA with Tukey’s test. *P < 0.05, **P < 0.01, ***P < 0.001

### W20/XD4-SPIONs rescued synapse loss in the brains of AD mice

The synaptic dysfunction and synapse loss correlate positively with cognitive decline in AD [18]. AβOs can impair synapse structure and function and lead to the decrease of synapse number. Postsynaptic density protein-95 (PSD-95) is the most abundant postsynaptic scaffolding protein in neurons [19]. Synaptophysin is a calcium-binding and integral membrane glycoprotein present in presynaptic vesicles in almost all neurons [20]. Both of these synaptic marker proteins play a key role in synapse development and plasticity. Here we evaluated the synaptic levels in mouse brains by immunohistochemistry using anti-PSD-95 and anti-synaptophysin antibodies, respectively (Fig. 6a, b). A significant decrease in both synaptic markers of PSD-95 and synaptophysin was detected in the cortex and hippocampus of AD mice compared with WT mice, while W20/XD4-SPIONs and W20-SPIONs significantly increased the levels of PSD-95 and synaptophysin in the cortex and hippocampus. XD4-SPIONs only increased synaptophysin levels (Fig. 6c). These findings suggested that W20/XD4-SPIONs significantly rescued synapse loss in the brains of AD mice.

**Fig. 6:** W20/XD4-SPIONs rescued synapse loss in the brains of AD mice. The PSD-95 immunostaining (**a**) and synaptophysin immunostaining (**b**) in the brains of WT and AD mice treated with various SPIONs. Scale bar 10 μm. (**c**) Quantification of PSD-95 and synaptophysin immunostaining in the cortex and hippocampal regions. n = 8 mice/group. Data represent means ± SEM and were analyzed by one-way ANOVA with Tukey’s test. *P < 0.05, **P < 0.01, ***P < 0.001

### W20/XD4-SPIONs enhanced Aβ engulfment by microglia in the brains of AD mice

To determine whether W20/XD4-SPIONs can promote Aβ engulfment by microglia in AD brains, the Aβ puncta in the Iba-1-positive microglia in mouse brains was qualified (Fig. 7a). We observed a significant increase in the microglial phagcytosis of Aβ in W20/XD4-SPIONs-treated AD mice compared with vehicle-treated AD controls. XD4-SPIONs and W20-SPIONs also resulted in a slight and significant increase in Aβ engulfment by microglia, but less than W20/XD4-SPIONs did (Fig. 7b).

**Fig. 7:** W20/XD4-SPIONs promoted microglial engulfment of Aβ in AD mice. **a** Representative images of Iba-1 positive microglia (green) and engulfed Aβ puncta (red) in WT and AD mice treated with various SPIONs. **b** Quantification of Aβ puncta engulfed in Iba-1 positive microglia, normalized to PBS-treated AD controls. Scale bars 500 nm. Data represent means ± SEM and were analyzed by one-way ANOVA with Tukey’s test. *P < 0.05, **P < 0.01, ***P < 0.001

## Discussion

Lots of clinical evidences revealed that AβOs, but not Aβ monomers and fibrils corelate well with AD dementia [10, 21]. Approaches targeting AβOs may have promising applications in AD treatment. The present work takes advantage of AβO-specific antibody W20 and SR-A activator XD4, when conjugated to SPIONs together, the obtained novel multifunctional nanoparticles W20/XD4-SPIONs can recognize AβOs and promote microglial phagocytosis of AβOs in the AD mouse brains. When administrated to a mouse model of AD for 28 days, W20/XD4-SPIONs rescued cognitive deficits and reduced neuropathology in AD mice. These findings indicated that W20/XD4-SPIONs had promising therapeutic potentials for AD upon early diagnostic value.

More than ten antibodies and vaccines targeting Aβ failed in the clinical trials. Most of these immunotherapies caused apparent side effects such as hydrocephalus, inflammation, amyloid-related imaging abnormalities with edema (ARIA-E), and ARIA-haemosiderin (ARIA-H) [22, 23], which were partly induced by complement-dependent cytotoxicity and microglial overactivation. The complex of Aβ and corresponding antibodies activated complement, producing proinflammatory fragments C3a and C5a. Also the resultant complement fragment such as C3b may further activate CR3 receptors of microglia, exacerbating neuroinflammation [24]. Therefore, the effector fragment of antibody plays a key role in the progression of side effects. ScFv antibody W20 is AβO-specific and without Fc fragment, which would eliminate associated adverse effects to a great extent.

However, W20 may reduce the microglial clearance of the complexes. To solve this problem, we further introduce the SR-A activator XD4 to the nanoparticles. Microglial phagocytosis and degradation of Aβ are believed to be the initial defense of the brains against toxic Aβ aggregates [25]. Multiple microglial cell surface receptors, including SR-A [26–28], class B scavenger receptor type I (SR-BI), CD36 [29], CD14, CD47 and toll-like receptors (TLRs), have been shown to mediate Aβ uptake and degradation [30]. With AD progression, microglia are overactivated and lack of intrinsic beneficial function of Aβ clearance, leading to Aβ accumulation, elevated levels of ROS and proinflammatory cytokines, neuroinflammation and neurodegeneration [31]. SR-A activation is beneficial for Aβ clearance and AD treatment. Compared with the activation of CR3 and Fcγ receptors, SR-A activation generated much less proinflammatory factors. Heptapeptide XD4 can activate SR-A on the glia by increasing the binding of Aβ to SR-A without the induction of proinflammatory cytokines, thereby promoting glial phagocytosis of Aβ and inhibiting Aβ-induced cytotoxicity [15]. In present study, W20/XD4-SPIONs retained XD4 property for SR-A activation, which significantly enhanced microglial engulfment of the AβOs recognized by W20, resulting in the pronounced improvement of cognitive performance in AD mice. W20/XD4-SPIONs containing these two safe components may exhibit good safety, which was confirmed by the present in vivo results that W20/XD4-SPIONs did not induce any adverse effects on cognitive function and neurophysiology in WT mice after 28 days of treatment (Figs. 3, 4, 5, 6).

In summary, besides the potential application in early diagnosis for AD, W20/XD4-SPIONs significantly rescued cognitive deficits, reduced Aβ burden and attenuated neuroinflammation, oxidative stress and synapse loss in AD mice. As W20/XD4-SPIONs contain both W20 and XD4, and possess dual therapeutic function, this kind of nanoparticles show the most beneficial effect on AD mice relative to W20-SPIONs or XD4-SPIONs, and exhibit promising therapeutic potentials for AD. However, the safety of W20/XD4-SPIONs should be thoroughly assessed using several kinds of animal models. Furthermore, a formal study of the pharmacokinetics of W20/XD4-SPIONs should be carried out to investigate the distribution and the half-life in brains.

## Methods

### Materials

Aβ42 and XD4 peptide were synthesized from Chinese Peptide Company (Hangzhou, China). Both Aβ40 and Aβ42 kits for Aβ measurement were purchased from Immuno-Biological Laboratories Co., Ltd. (Gunma, Japan). TNF-α, IL-1β and IL-6 ELISA kits were obtained from Neobioscience Technology Co., Ltd. (Beijing, China). The following antibodies were used: 6E10 (monoclonal raised against Aβ1-16, Signet, SIG39300), W20 (oligomer-specific antibody, developed and prepared in our laboratory), anti-Iba-1 antibody (GenTex, GTX100042), anti-GFAP antibody (Abcam, ab53554), anti-PSD-95 antibody (Abcam, ab18258), anti-synaptophysin antibody (Abcam, ab32127), anti-COX2 antibody (Abcam, ab179800), anti-iNOS antibody (Abcam, ab178945), anti-GAPDH antibody (CST, 2118S), goat anti-rabbit secondary antibody conjugated to Alexa Fluor 488 (Santa Cruz, I1112) or Alexa Fluor 594 (Abcam, ab150084), HRP-conjugated goat anti-mouse or rabbit IgG antibody (Zhongshan Golden Bridge Biotechnology, Beijing, China).

### Preparation of W20 and/or XD4 conjugated-SPIONs

W20 and/or XD4 conjugated-SPIONs were synthesized according to previous methods [16]. Briefly, the PEG-coated SPIONs were synthesized by a “one-pot” synthetic approach. 2.1 g of Fe(acac)_3_, 7.9 mL of oleylamine, and 24 g of HOOC-PEG-COOH (Mn = 2000) were dissolved in 100 mL of diphenyl ether solution and incubated at 80 ℃ for 4 h with stirring at 400 rpm in anaerobic environment, then the PEG-SPIONs were precipitated by ether and dissolved in PBS for further experiments. Two mg PEG-SPIONs were mixed with 2.50 μmol EDC and 6.25 μmol sulfo-NHS in 950 μL PBS buffer and incubated for 15 min at room temperature. Then 1 mg W20 and/or 0.1 mg XD4 (in 50 μL of PBS) were added and the reaction was undergoing overnight at 4 °C. The resultant conjugated-SPIONs were collected by centrifugation at 25,000 rpm and kept at 4 °C for future use. The conjugative efficiency for W20 or XD4 was calculated by determining the residual protein amount in the supernatant using BCA assay. The supernatant was transferred to a 3 kD ultrafiltration tube and centrifuged for 15 min. The protein amount in the filtrate fraction was measured as the residual XD4, and proteins in the cut-off solution can be determined as the residual W20. The conjugative efficiency was calculated according to the following equation:

$${\text{Conjugation }}\left( {\text{\%}} \right) = \frac{{{\text{total added W}}20{\text{ or XD}}4 - {\text{ W}}20{\text{ or XD}}4{\text{ in supernatant}}}}{{{\text{total added W}}20{\text{ or XD}}4}} \times 100{ }{\text{.}}$$

### Nanoparticle characterization

The hydrodynamic size of the nanoparticles was characterized by DLS using Zetasizer Nano ZSP (Malvern, UK) at room temperature. TEM was used for the morphological examination of the nanoparticles operating at an accelerating voltage of 100 kV (HITACHI, HT7700, Japan). More than 100 quasi-spherical particles were measured to determine the average diameters of the nanoparticles.

### Nanoparticle biodistribution

Various SPIONs were conjugated to fluorescent dyes using a Cy7 Labeling Kit (FANBO biochemicals, CAT#1060). The Cy7-labeled SPIONs were separated by using a 10 kD ultrafiltration tube to remove excess dye. Five-week-old male nude mice were injected with 300 μL Cy7-labeled nanoparticles (200 μmol Fe/kg body weight) intravenously via the tail vein in combination with or without 15% mannitol. The mice were sacrificed at 6 h post administration after heart perfusion with ice-cold PBS containing heparin (10 U/mL). Their brains were collected, and the specific Cy7 fluorescence was quantified using the IVIS Spectrum imaging system (Kodak In-Vivo Imaging System FX Pro, USA).

### Thioflavin T fluorescence assay

To determine the effects of W20/XD4-SPIONs and W20-SPIONs on Aβ42 aggregation, 10 μM Aβ42 was mixed with 100 μg/mL or 1000 μg/mL of SPIONs and incubated at 37 °C without agitation. When monitoring the aggregation kinetics of Aβ42, a 10 μL aliquot of sample was mixed with 190 μL Th T solution (5 μM), and the Th T fluorescence intensity was measured using a Tecan Safire2 microplate reader (Tecan, Switzerland) set to 450 nm/482 nm (excitation/emission). Data were obtained from three independent experiments.

### MTT assay

SH-SY5Y cells (obtained from the cell line resource center of Peking Union Medical College, Chinese Academy of Medical Sciences) were maintained in Dulbecco’s modified Eagle’s medium (DMEM; Hyclone) with 10% fetal bovine serum (FBS) and 1% penicillin/streptomycin at 37 °C under a 5% CO_2_ atmosphere. The cells were seeded in 96-well plates with approximately 10,000 cells per 100 μL of medium per well. Plates were then incubated at 37 °C for 24 h to allow cells to attach. The SPIONs with or without 4 μM Aβ42 oligomers were added to the wells and then incubated for an additional 48 h at 37 °C. Cell viability was determined by adding 20 μL of 5 mg/mL MTT to each well. After 3 h of incubation at 37 °C, the supernatants were replaced with a 150 μL aliquot of DMSO in the dark. The absorbance at 570/630 nm was measured by using a SpectraMax M5 microplate reader (Molecular Devices, Sunnyvale, CA, USA). Data were obtained from three independent experiments.

### Measurements for proinflammatory cytokines

BV-2 cells (obtained from the cell line resource center of Peking Union Medical College, Chinese Academy of Medical Sciences) were maintained in DMEM with 10% FBS and 1% penicillin/streptomycin at 37 °C in 5% CO_2_. The cells were treated with various SPIONs with or without 4 μM Aβ42 oligomers and incubated for 12 h at 37 °C. Then the cell supernatants were collected and the levels of TNF-α and IL-6 were determined using ELISA kits (Neobioscience technology, Beijing, China) according to the manufacturer’s protocols. Briefly, the cell supernatants were added to a 96-well ELISA plate and reacted with the relevant primary antibodies followed by HRP-conjugated secondary antibodies. 3,3,5,5-Tetramethylbenzidine was used as the substrate. The absorbance of the samples was measured at 450 nm using a SpectraMax M5 microplate reader (Molecular Devices, Sunnyvale, CA, USA). Data were obtained from three independent experiments.

### Western blot analysis

Proteins samples from BV-2 cell lysates pretreated with 4 μM Aβ42 oligomers and various SPIONs were separated by 12% SDS-PAGE gel (Invitrogen) and transferred onto nitrocellulose membrane (Merck Millipore). After blocking with 5% nonfat milk for 1 h at room temperature, the membrane was probed with anti-iNOS (1:1000), anti-COX2 (1:1000) and anti-GAPDH (1:1000) antibodies respectively, and followed by appropriate HPR-conjugated secondary antibodies. Bands in immunoblots were developed with Super-Signal West Pico Plus Chemiluminescent Substrate kit (Pierce, UB278521), and quantified by densitometry using ImageJ software (National Institutes of Health, NIH, USA).

### Animal treatment

APPswe/PS1dE9 transgenic mice were obtained from the Jackson Laboratory. All mice were given food and water ad libitum and maintained in a colony room at 22 ± 2℃ with 45% ± 10% humidity under a 12:12 h light/dark cycle. Six-month old male AD mice were categorized into five groups: PBS-treated (AD-PBS, n = 8), SPIONs-treated (AD-SPIONs, n = 8), XD4-SPIONs-treated (AD-XD4-SPIONs, n = 8), W20-SPIONs-treated (AD-W20-SPIONs, n = 8) and W20/XD4-SPIONs-treated (AD-W20/XD4-SPIONs, n = 8), and their WT littermates were categorized into three groups: PBS-treated (WT-PBS, n = 8), SPIONs-treated (WT-SPIONs, n = 8) and W20/XD4-SPIONs-treated (WT-W20/XD4-SPIONs, n = 8). The mice were administered with a daily dose of 1 mg nanoparticles in 100 μL PBS (0.01 M, pH 7.4) with 15% mannitol via tail vein for 28 days. After the last administration, the behavioral tests were performed.

### Y-maze test

The Y-maze test consisted of two trials separated by an interval of 1 h. The first trial was 10 min in duration and allowed the mouse to explore only two arms (the start and familiar arms) of the maze, with the third arm (novel arm) blocked. In the second trial, the mouse was put in the same starting arm as in trial 1 with free access to all 3 arms for 5 min. The total time spent and the number of entries in the novel arm were video recorded and analyzed. The arms were cleaned with 70% alcohol between trials to eliminate olfactory cues.

### Morris water maze test

The water maze consisted of a pool (110 cm in diameter) containing opaque water (22 ± 1 °C) and a platform (10 cm in diameter) submerged 1 cm under the water. Hidden platform training was carried out twice per day over five consecutive days, with an inter-trial interval of 3–4 h. Mice were allowed to swim for 60 s to find the platform, on which they were allowed to stay for 10 s. The trial ended when the mouse located the platform. Mice unable to locate the platform were guided to it. 24 h after the acquisition trial, the mice were tested for memory retention in a probe trial in the absence of the hidden platform. The performance of each mouse was monitored using a video camera (Sony, Tokyo, Japan) mounted over the maze and automatically recorded via a video tracking system.

### Object recognition test

The object recognition test was performed as previously described with slight modifications [32]. Briefly, in the habituation phase, mice were allowed to freely explore the behavioral open-field arena (50 cm × 50 cm × 25 cm white plastic box, empty) individually for 5 min one day before the test. For the training session (Trial 1), mice were allowed to explore for 5 min in the same box having two identical objects in the upper two corners. For the testing session (Trial 2), after a 24 h retention period, the object in the right corner was replaced with a novel object, and the mice were reintroduced to the box and allowed to explore for 5 min. Time spent exploring and sniffing each object was recorded. The results are expressed as the discrimination index by calculating: $\frac{Time novel - Time familiar}{{Time novel + Time familiar}} \times 100 \left( \% \right)$. The box was cleaned with 70% alcohol between tests to eliminate olfactory cues.

### Immunohistochemistry

Mice were deeply anaesthetized with avertin (250 mg/kg) and transcardially perfused with ice-old PBS containing heparin (10 U/mL) before sacrificed. Their brains were immediately removed and divided along the sagittal plane. The left brain hemisphere was fixed in 4% paraformaldehyde at 4 °C overnight and processed for paraffin-embedded sections. Coronal paraffin-embedded serial sections of 5 μm thickness were cut on a Lecia CM1850 microtome (Leica Biosystems, Buffalo Grove, IL, USA). For immunohistochemistry analysis, sections were deparaffinized and subjected to antigen retrieval using citrate buffer (0.01 M, pH 6.0, 0.05% Tween-20) in a steamer at 95 °C for 20 min. The sections were then incubated with 3% H_2_O_2_ to quench endogenous peroxidases and washed 3 times with 1 × PBST. Thereafter, sections were permeabilized and blocked with 10% normal goat serum in 0.3% Triton X-100 PBST for 1 h at room temperature. Subsequently, the sections were incubated with 6E10 (1:100), anti-Iba-1 (1:100) and anti-GFAP (1:100) antibodies, respectively, followed by corresponding HRP-labeled secondary antibody and visualized with diaminobenzidine (DAB). For synaptophysin and PSD-95 staining, sections were immunostained with anti-synaptophysin (1:100) and anti-PSD95 (1:100) antibodies followed by corresponding secondary antibody conjugated to Alexa Fluor 488 (1:200). All images were acquired with an Olympus IX73 inverted microscope with DP80 camera. For immunostaining quantification, four coronal sections spanning the cortex and hippocampus at different depths were analyzed for each animal. Six images were acquired on matching areas of each cortex and hippocampus per section. Values from each section were averaged to obtain a mean value for each animal. The values obtained for each mouse group were averaged. Aβ deposits were presented as the per cent area occupied by 6E10-immunoreactive deposits. For the other immunostaining analysis, the data were normalized to the mean value of WT or vehicle-treated AD control mice and expressed as percentage means ± SEM. All images were processed and analyzed by ImageJ Software.

For microglia engulfment analysis, paraffin-embedded sections of 20 μm thickness were immunostained for Aβ with 6E10 (1:100) and microglia marker with anti-Iba-1 antibody (1:100) followed by corresponding secondary antibody conjugated to Alexa Fluor 594 (1:200) and Alexa Fluor 488 (1:200), respectively. The brain sections were imaged on a Leica TCS SP8 confocal microscope. The Aβ puncta engulfed by the Iba-1-positive microglia were quantified. 8–10 microglia cells were analyzed per mouse.

### Brain lysate preparation

The right brain hemisphere was homogenized in RIPA buffer containing protease inhibitor cocktail (Sigma, P2714-1BTL). The tissues were then centrifuged at 14,000×*g* for 30 min at 4 °C, and the supernatant (RIPA-soluble fraction) containing soluble Aβ was collected. The pellets were resuspended in guanidine buffer (5.0 M guanidine-HCl/50 mM Tris–HCl, pH 8.0) and centrifuged at 14,000×*g* for 1 h at 4 °C to obtain supernatants containing insoluble Aβ (guanidine-soluble fraction).

### Measurements for Aβ and proinflammatory cytokines in the brain lysates

The levels of RIPA-soluble Aβ and RIPA-insoluble (guanidine-soluble) Aβ in the brain lysates of mice were quantified by ELISA using Aβ40 and Aβ42 immunoassay kits (Immuno-Biological Laboratories). For the proinflammatory cytokine measurements, the levels of TNF-α, IL-1β and IL-6 in the brain lysates of mice were determined using corresponding ELISA kits (Neobioscience Technology) according to the manufacturer’s protocols.

### Measurement of GSH, GSSG and ROS

The levels of GSH and GSSG in the brain lysates were assayed by commercial kits (Beyotime, S0053). Total GSH was measured by 5,5-dithiobis (2-nitrobenzoic) acid (DTNB)-GSSG reductase recycling. GSSG was obtained by determining the absorbance of 5-thio-2-nitrobenzoic acid produced from the reaction of the reduced GSH with DTNB according to the manufacturer’s protocols. The reduced GSH was obtained by subtracting GSSG from the total GSH. The absorbance was determined at 412 nm by using an MD-M5 microplate reader.

ROS assay was performed as previously described [33]. Briefly, ROS production was fluorometrically monitored using 2,7-dichlorofluorescein diacetate (DCFDA) mixed with the brain lysates. The intensity of DCF fluorescence generated from carboxy-DCFDA was proportional to the amount of ROS. The fluorescence was determined using an MD-M5 microplate reader (excitation, 485 nm; emission, 530 nm) and the ROS units were calculated.

### Statistical analysis

Data were analyzed with GraphPad Prism v.8. Statistical significance was assessed using one-way ANOVA followed by Tukey’s test, or two-way ANOVA followed by Dunnett’s test, as appropriate. Results were expressed as group mean ± SEM, and P < 0.05 was considered statistically significant. All samples or animals were included for statistical analysis unless otherwise noted in pre-established criteria.

## Data Availability

All data associated with this study are available in the main text.
